This article has been retracted.

# 5G Massive MIMO Signal Detection Algorithm Based on Deep Learning

**DOI:** 10.1155/2022/9999951

**Published:** 2022-02-27

**Authors:** Lichao Yan, Yi Wang, Ning Zheng

**Affiliations:** School of Intelligent Engineering, Zhengzhou University of Aeronautics, Zhengzhou, Henan 450046, China

## Abstract

Aiming at the problems of poor signal detection effect caused by many interference factors in large-scale MIMO technology scene, this paper proposes a 5G massive MIMO signal detection algorithm based on deep learning. Firstly, the MIMO system model based on neural network is constructed, and Deep Neural Network (DNN) detection is introduced into the receiver of the traditional MIMO system to obtain the information bits or codewords and channel state information transmitted by transmitters. Then, the end-to-end training method is adopted to make neural network learn the mapping relationship of information bits or codewords transmitted by system transceivers. Furthermore, DNN detector is improved based on Simplified Message Passing Detection (sMPD) algorithm, and the correction factor is updated continuously to optimize network parameters to realize the accurate detection and decoding of the MIMO system. Finally, the proposed algorithm is experimentally analyzed based on the TensorFlow deep learning framework. Experimental results show that when signal-to-noise ratio is 10 dB, the bit error rate and mean square error are lower than 0.005 and 0.1, respectively.

## 1. Introduction

At present, as one of mainstream research directions in the field of wireless communication, intelligent communication is actively introducing artificial intelligence technology into all levels of the wireless communication system, which has become an effective way to explore the field of intelligent communication [1]. As one of key technologies of the 5G mobile communication system, large-scale Multiple Input Multiple Output (MIMO) technology has high spectrum utilization and link reliability [2]. However, due to the increase in number of antennas configured at transceiver end of the MIMO system, the signal processing process at receiving end of the communication system becomes more complicated, which will make signal detection face a huge challenge of high computational complexity [3, 4]. Therefore, designing signal detection algorithms with low computational complexity and high detection performance is an urgent problem for massive MIMO systems [5]. The popular research direction of the MIMO system has turned to the suboptimal detection algorithm.

The purpose of massive MIMO signal detection is to recover the original signal at the transmitter under noise and interference environments. It is an important link to improve the overall performance of the system and reduce the complexity of the system [6]. Low-complexity signal detection algorithms have become a research hotspot in recent years [7]. For classic linear detection algorithms such as ZF detection, the computational complexity is too high due to its large number of matrix inversion operations [8], the detection performance of linear detection algorithm is not ideal, so it is difficult to apply to the actual massive MIMO system [9]. Reference [10] proposed a low-complexity massive MIMO detection method based on approximate expected propagation. This method uses the approximation method of the channel hardening phenomenon to eliminate matrix inversion during iteration and reduces the computational complexity of accurate detection while maintaining good performance. In reference [11], a linear detector based on conjugate gradient of multiple search directions was proposed in the massive MIMO uplink system in order to reduce the complexity of data detection. It determined the search direction in each subdomain by the projection method, which improves the performance of the algorithm. However, the loop effect caused problems such as slow or nonconvergence, which leads to a decrease in algorithm detection performance. Reference [12] proposed a system model that considers the reverberation effect of radar systems on massive MIMO receivers using the receiver for uplink to perform channel estimation and data detection. The experimental results proved the effectiveness of the proposed detection scheme. Reference [13] proposed an iterative precoding scheme based on Chebyshev acceleration. The simulation results showed that the proposed method has lower complexity while ensuring higher detection performance. However, it was difficult to be widely used in actual promotion and application due to the limitations of the coding scheme.

As deep learning has made great achievements in other fields, there are more and more research studies on applying deep learning to communication systems [14]. Orthogonal approximation message passing detection neural network uses the idea of the orthogonal approximation message passing detection algorithm, while increasing adjustable parameters using deep learning optimization methods to improve its detection performance. Reference [15] proposed a heuristic method for pilot/data power optimization. This method could improve algorithm performance through space-time block coding when the access point does not have any channel state information. However, when applied to a high-order modulation system, the computational complexity will increase as the number of users and modulation order increase. Reference [16] algorithm could speed up the convergence speed by reducing the spectral radius of the rederived iterative matrix. Reference [17] proposed a MIMO detection scheme based on deep learning using a novel training algorithm. The algorithm accelerated the training by time and spectrum correlation in the real channel, so that it has lower computational complexity than the existing methods on real channel. However, each neural network layer needs to perform matrix inversion operation, which brings high computational complexity. The computational advantages of deep learning improve the detection performance of massive MIMO signals. However, the method of extending the iterative algorithm to neural network is more dependent on the channel environment [18].

This paper proposes a massive MIMO signal detection algorithm based on deep learning to address the problems of large number of MIMO antennas in the 5G communication system, which makes signal detection difficult. Compared with traditional detection algorithms, its innovations are summarized as follows:

1. Due to the complexity of DNN parameters, the proposed algorithm uses the Simplified Message Passing Detector (sMPD) algorithm to optimize network parameters iteratively to reduce the computational difficulty and improve network signal analysis capabilities.
2. In order to realize the accurate detection of massive MIMO signal, the proposed algorithm constructs a detection system based on neural network. Among them, DNN detector improved by the sMPD algorithm is used to analyze MIMO signal to achieve low error signal transmission.

## 2. System Model and Problem Analysis

Consider a massive MIMO system in a single-cell multiuser Time Division Duplex (TDD) mode. The base station is equipped with *M* antennas, and the uplink channel estimation process is shown in Figure 1.

In the uplink, the base station receives signals simultaneously transmitted by *N* single antenna user in the same time-frequency resource, which can be expressed as follows:

(1) $$\begin{array}{c} y\left(t\right)=\mathrm{Gx}\left(t\right)+\delta \left(t\right), \end{array}$$

where **G** represents the flat fading channel matrix of *M* × *N* between the base station and *N* users, **x**(*t*) represents the signal vector of *N* × 1 sent by *N* users at time, and *δ*(*t*) represents additive white Gaussian noise with a mean value of 0 and a variance of *σ*_*n*_^2^/2.

Assuming that each user transmits an orthogonal pilot sequence of length *L*(*L* ≥ *N*) in the channel coherence time, the pilot signal matrix received by base station is as follows:

(2) $$\begin{array}{c} \mathrm{Y=G\Psi +,}\hat{\delta } \end{array}$$

where Ψ=[*φ*(1), *φ*(2), ⋯, *φ*(*L*)] is the pilot matrix of dimension *N* × *L* that contains all user training sequences and $\hat{\delta }$ is an additive white Gaussian noise matrix whose elements are all Gaussian random variables with independent identically distributed mean value 0 and variance *σ*_*n*_^2^/2.

According to the system model, Rice flat fading channel matrix **G** can be further expressed as follows:

(3) $$\begin{array}{c} G=\sqrt{\frac{\kappa }{\kappa +1}}\bar{G}+\sqrt{\frac{1}{\kappa +1}}\tilde{G}\text{,} \end{array}$$

where $\bar{G}$ represents the deterministic component matrix containing line-of-sight signal and $\tilde{G}$ represents Rayleigh random component matrix containing the scattered signal. *κ* ≥ 0 is the Rice fading factor; when *κ*=0, the channel is Rayleigh channel, that is, $\mathrm{G=}\tilde{G}$.

For the deterministic component $\bar{G}$, it can be expressed as

(4) $$\begin{array}{c} {\left[\bar{G}\right]}_{mn}=e^{-j\left(m-1\right)\frac{2\pi d}{\lambda }\sin\left(\theta_{n}\right)}, \end{array}$$

*d* and *λ* represent the base station antenna spacing and radio wave wavelength, respectively, and *θ*_*n*_ represents the angle of arrival of *n* user.

For Rayleigh random component $\tilde{G}$ containing the scattered signal, the finite scattering channel model is considered. Assuming that each user has *q* paths to base station, the channel vector **g**_*n*_ from the *n* user to the base station can be expressed as follows:

(5) $$\begin{array}{c} \;g_{n}=\frac{1}{\sqrt{Q}}\sum_{q=1}^{Q}h_{nq}\phi \left(\theta_{q}\right)\\ \phi \left(\theta_{q}\right)={\left[1,e^{-j2\pi d/\lambda \cos\left(\theta_{q}\right)},\cdots ,e^{-j2\pi \frac{\left(M-1\right)d}{\lambda }\cos\left(\theta_{q}\right)}\right]}^{T}, \end{array}$$

where *h*_*nq*_ is the random transmission gain of *q* path. In order to facilitate the analysis without loss of generality, it is assumed that the path gain obeys a complex Gaussian distribution with a mean value of 0 and a variance of 1. *θ*_*q*_ is the random arrival angle of *q* path; *ϕ*(*θ*_*q*_) is the direction vector under ULA model; and *d* and *λ* represent the base station antenna spacing and radio wave wavelength, respectively.

In the massive MIMO system, it is usually relevant on the base station side but not on the user side. This is due to the limited number of scatterers on base station side, while the users have relatively abundant scatterers [19, 20]. Therefore, it can be assumed that the antenna direction vectors of users are the same, and the random component channel matrix can be expressed as follows:

(6) $$\begin{array}{c} \mathrm{G=\Omega}\tilde{H}, \end{array}$$

where Ω=[*ϕ*(*θ*_1_), *ϕ*(*θ*_2_),…, *ϕ*(*θ*_*q*_)] is the full-rank matrix of *M* × *Q* containing *Q* direction vectors; **H** is the path gain matrix of *Q* × *N*; [**H**]_*q*.*n*_=*h*_*nq*_.

According to the nature of rank, in Rice flat fading channel model, the rank of **G** is $\text{rank}\left(G\right)\leq \text{rank}\left(\bar{G}\right)+\text{rank}\left(\tilde{G}\right)$. The number of antennas *M* and the number of users *N* are usually large (*M* ≫ *N*), while the number of effective paths *Q* is relatively small. Therefore, in the physical finite scattering model, the rank $\text{rank}\left(\tilde{G}\right)=\min\left\{M,N,Q\right\}=Q$ of Rayleigh random component $\tilde{G}$. The rank rank(**G**) ≤ *N*+*Q* of channel matrix **G** is significantly smaller than the matrix dimension.

## 3. MIMO Signal Detection Model Based on Neural Network

### 3.1. MIMO System Model

Taking the MIMO system as the main research object, *M*_*t*_ and *M*_*r*_ antennas are installed in the transceiver end of the system. The model structure of the MIMO communication system is shown in Figure 2. In order to accurately detect and decode the transmitted information at the receiving end of MIMO system, aiming at this goal, it mainly combines DNN and autoencoder neural network model. The two different neural network structures and physical layer framework of the traditional MIMO wireless communication system are organically integrated. Its purpose is to process the information bits or code words received by the MIMO system.

The mathematical model of the entire MIMO system can be expressed by the following linear equation:

(7) $$\begin{array}{c} \mathrm{y=Gx+\delta ,} \end{array}$$

where **x**=[*x*,…,*x*_*M*_*t*__]^*T*^ ∈ *ℂ*^*M*_*t*_×1^ represents the information vector sent by the transmitting end of the system and **y**=[*y*_1_,…,*y*_*M*_*r*__]^*T*^ ∈ *ℂ*^*M*_*r*_×1^ is the information vector received by the receiving end of the MIMO system.

### 3.2. Input and Output of Neural Network

The number of neurons in input layer of a neural network generally depends on the attributes of sample data. In the proposed neural network model, matrix **G** and vector **y** are used as the input of neural network. Before input, the data are preprocessed, matrix **G** is converted into a (*M* × *N*) dimensional column vector, and the column vector is combined with column vector **y**. Since each element of column vector is a complex number, the real part and the imaginary part are separated and connected in series as the network input **I**, **I**=[*g*_1,1_, *g*_2,1_,…,*g*_*M*,*N*_, *y*_1_, *y*_2_,…,*y*_*M*_]^*T*^. The number of input neurons of neural network is 2(*N* × *M*+*M*), and the activation function of output layer is selected according to digital modulation mode of the MIMO system [21]. Taking binary phase shift keying as an example, since the transmitted signal symbol is 0 or 1, the activation function is selected as Sigmoid function. The reason is that the output of Sigmoid is mapped in the range of (0, 1), which has a strong correlation with the transmitted symbol. For the modulation method, a linear activation function can be selected [22]. After neural network is output, the output is recombined into the transmission signal pattern, and symbol decision is performed, and the result is detection signal *x*^*∗*^ of MIMO system receiver based on neural network. The flow of entire data in the receiver is shown in Figure 3.

### 3.3. Designed DNN Detector Based on sMPD Algorithm

A detection network is designed based on the sMPD algorithm, which relies on the sMPD algorithm. That is, using the existing algorithm as a starting point, each iteration of the sMPD algorithm is expanded to each layer in the network, and the optimization method of deep learning is used to obtain the best training parameters to obtain a neural network that meets the signal detection performance requirements [23, 24]. From this perspective, deep learning provides a powerful tool. It can make the improved MPD get the best correction factor to achieve higher performance. In addition, DNN detector designed based on the sMPD algorithm constructs a DNN by expanding each iteration of iterative sMPD to each layer of detection network. Among them, correction factor set is the parameters to be optimized, and the best correction factor is obtained by “learning” by deep learning training [25].

DNN is one of typical deep learning models, which can map input *x*_0_ ∈ *ℂ*^*M*_*t*_×1^ to output *y*_0_ ∈ *ℂ*^*M*_*r*_×1^:

(8) $$\begin{array}{c} y=f\left(x_{0},\varpi \right), \end{array}$$

where *ϖ* represents the parameter that approximates optimal function, which maps the input to desired output.

DNN usually has multiple hidden layers between the input and output layers, and a multilayer neural network combines many functional units. For a DNN with *K* layers, the output of (*k* − 1) is used as the input of *k* layer, and the mapping function of *k* layer can be defined as follows:

(9) $$\begin{array}{c} x_{k}=f^{\left(1\right)}\left(x_{k-1};\varpi_{k}\right), \end{array}$$

where *ϖ*_*k*_ represents the training parameters of the *k* layer and *f*^(1)^(*x*_*k*−1_; *ϖ*_*k*_) is the mapping function of the *k* layer.

Due to the similarity of the factor graph model and DNN structure, DNN can be designed by unfolding iterative algorithm. Each iteration in the algorithm corresponds to each layer in the network, as shown in Table 1. The comparison of MPD's factor graph model and DNN structure confirms that they have similar structures. Based on a reasonable design of detection network, the MPD algorithm can be further improved through the optimization method of deep learning.

In the damped MPD algorithm, the damping factor for each iteration can be different. When selecting the normalization/offset factors of sMPD, these factors can be expanded to have a different symbol probability *p*_*ij*_^(*k*)^ for each message. In fact, a different correction factor can be set for each message in each iteration, and the calculation of prior probability can be expressed in a unified manner. Specifically, by increasing the damping factor, *p*_*ij*_^(*k*)^ is defined as follows:

(10) $$\begin{array}{c} p_{ij}^{\left(k\right)}⇐\left(1-\beta_{ij}^{\left(k\right)}\right)p_{ij}^{\left(k\right)}+\beta_{ij}^{\left(k\right)}p_{ij}^{\left(k-1\right)}, \end{array}$$

where *β*_*ij*_^(*k*)^ is the weighted average damping factor of message calculated in the current iteration and the message obtained in the previous iteration.

To further increase the correction factor *τ*_*ij*_^(*k*)^ and bias factor *μ*_*ij*_^(*k*)^, (10) is converted to the following:

(11) $$\begin{array}{c} p_{j}^{\left(k\right)}⇐\left(1-\beta_{j}^{\left(k\right)}\right)\left(\tau_{ij}^{\left(k\right)}p_{ij}^{\left(k\right)}-\mu_{ij}^{\left(k\right)}\right)+\beta_{ij}^{\left(k\right)}p_{ij}^{\left(k-1\right)}. \end{array}$$

The damped sMPD algorithm requires multidimensional parameters to approximate MPD, and these multidimensional parameters are designed to further improve performance. However, it will lead to an increase in the number of parameters to be optimized, especially when the number of transmitting and receiving antennas is large. For traditional methods, this is a complex optimization problem. However, it can be solved by deep learning, a powerful optimization tool [26].

In summary, the first iteration of the improved MPD algorithm can be summarized by two kinds of messages, including Log-Likelihood Ratio (LLR) *ζ*^(*k*)^ and probability *p*^(*k*)^ and the set of correction factor *τ*^(*k*)^. A complete iteration in the sMPD algorithm can be mapped to a layer in DNN to construct DNN-MIMO detector and use *τ*^(*k*)^ as the training parameter set to be learned. Specifically, the DNN detector based on sMPD is expressed as follows:

(12) $$\begin{array}{c} \left\{\begin{array}{c} \zeta^{\left(k\right)},p^{\left(k\right)}=f^{\left(k\right)}\left(\zeta^{\left(k-1\right)},p^{\left(k-1\right)},\tau^{\left(k\right)}\right)\\ o=\sigma \left(\zeta^{\left(K\right)}\right) \end{array}\right., \end{array}$$

where *f*^(*k*)^(*ζ*^(*k* − 1)^, *p*^(*k* − 1)^, *τ*^(*k*)^) is the mapping relationship of *l*-th iteration in the improved MPD algorithm, *o* is the final output of DNN, and *σ*(·) is the normalization function. The output *ζ*^(*K*)^ of the *K* final iteration is rescaled within the range of [0, 1].

For the sMPD algorithm, *ζ*^(*k*)^={*ζ*_*j*_^(*k*)^} and *p*^(*k*)^={*p*_*j*_^(*k*)^}, and training factor Δ={*α*^(1)^,…, *α*^(*K*)^, *ω*^(1)^,…, *ω*^(*K*)^, *b*^(1)^,…, *b*^(*K*)^} include attenuation, scaling, and bias factors. This sMPD-based DNN detector is called an Improved MPD (IMPD). The overall structure of IMPD detector is shown in Figure 4. The hidden layer in DNN is expanded by the sMPD algorithm. These hidden layers are also different according to the iterative process of the selected MPD algorithm, thus forming a variety of different DNN detectors.

In order to measure the detection performance of signal detection network designed for the massive MIMO system, cross entropy is used to express the error between output of neural network and real transmitted signal. And the minimum SGD method is used to minimize loss function to determine the best correction factor set (Δ).

The IMPD detector includes two stages of learning and detection. First, neural network is trained to obtain the optimized correction factor. After that, trained DNN detector is used for signal detection. This DNN based on MPD training is similar to the MPD algorithm, except that the optimized correction factor is obtained through the training process. Therefore, IMPD detector can be regarded as a special case of the MPD algorithm and requires additional training preprocessing. However, this is all done offline on the computer, and it will not increase the complexity of performing real-time detection tasks.

### 3.4. Batch Normalization and Dropout

The proposed neural network model is relatively complicated, and there are too many parameters that need to be updated, so it is prone to overfitting during the training process. Overfitting means that the function fitted by the neural network fits the training set perfectly, but the results of validation set and test set containing new data are poor. That is, the training data are overfitted without considering the generalization ability of network.

The overfitting phenomenon can be solved by batch normalization and dropout. Batch training refers to training a batch of data at a time during the neural network training process. The purpose of training is to reduce the loss function value of entire batch of data. This can reduce the randomness caused by a single data training as much as possible. A batch of data is called a batch, and all training sets the batch value to 1000. Dropout was first proposed by Hinton in 2012. It refers to randomly ignoring a certain percentage of neurons during neural network training. The neural network model using Dropout randomly selects a certain number of neurons for training during the training process and does not need to rely too much on certain local features. This can reduce the interaction between feature detectors (neurons) and make the model more generalized. Using Dropout in the training process is equivalent to different neural networks for each training, and each neural network will also give different results. However, as the training process progresses, most of neural network output results will be correct. Then, a small number of wrong results will not affect the total output. The Dropout operation was used during training.

## 4. Experiment and Analysis

With the help of advanced deep learning libraries such as TensorFlow, the proposed algorithm is experimentally analyzed, and the simulation parameter settings are shown in Table 2.

### 4.1. Performance Comparison of Deep Learning and Linear Detection Algorithms

The performance of the used deep learning method is compared with that of the traditional linear detection algorithm (maximum likelihood algorithm and zero-forcing algorithm). The result of bit error rate (BER) is shown in Figure 5.

It can be seen from Figure 5 that the detection performance based on the deep learning method applied to MIMO system signal detection is lower than the performance of the optimal maximum likelihood detection algorithm. However, it is significantly better than zero-forcing detection algorithm performance. Since the principle of the traditional linear detection algorithm is relatively simple, the proposed algorithm shows better performance advantages after testing the neural network with better training effect. When BER is 0.01, signal-to-noise ratio (SNR) difference between the deep learning method and maximum likelihood detection algorithm is about 2.5 dB. BER is in the range of 0.1 to 0.01. This deep learning method has a performance gain of nearly 2 dB.

### 4.2. Performance Comparison of Deep Learning and Belief Propagation Decoding Algorithms

In order to further verify the performance of the deep learning method in channel decoding in the MIMO communication system, the decoding performance of the Back Propagation (BP) algorithm of polarization code is selected and compared. In the experiment, the number of iterative cycles of the BP decoding algorithm is set to 200. After the iteration loop, the BER result obtained is shown in Figure 6.

It can be seen from Figure 6 that the performance of channel decoding based on deep learning is better than that of the traditional BP decoding algorithm. When BER is 0.01, the decoding method using autoencoder neural network has a performance gain of about 1.5 dB. The decoding performance of DNN also has a performance gain of nearly 1 dB. This demonstrates that the deep learning method can improve channel decoding performance of the MIMO system.

### 4.3. Detection Performance Comparison of Different Algorithms

In order to demonstrate the performance of the proposed algorithm, the algorithms in reference [11], reference [13], and reference [16] are compared In SNR range of 0∼10 dB, the trained model will be tested, and BER results under different SNRs are shown in Figure 7.

It can be seen from Figure 7 that in the same SNR range, the detection performance of the proposed algorithm is better than that of other comparison algorithms. When SNR is 10 dB, its BER is lower than 0.005. because the proposed algorithm constructs a detection system based on neural network and uses the DNN detector improved by the sMPD algorithm to analyze MIMO signals, so low error signal transmission is realized. The improved linear detection algorithm used in reference [11] is affected by loop effect, and its detection performance is not good. When SNR is 9 dB, its BER is still higher than 0.01. Reference [16] carried out parallel iteration based on the linear detection algorithm, and the detection speed and performance have been improved to a certain extent. However, the data processing capability of the linear detection algorithm itself is insufficient, so there is a significant gap compared with IMPD of the proposed algorithm. Reference [13] used the iterative precoding algorithm of Chebyshev acceleration for signal detection. Only from the iterative aspect of optimization, its detection performance improvement effect is not obvious. Thus, when BER is 0.01, the detection performance of the proposed algorithm and reference [13] had a performance gain of nearly 1.5 dB. And within this SNR range, the detection performance of the MIMO system shows the most obvious advantages.

Besides, mean square error (MSE) results of four comparison algorithms under different SNRs are shown in Figure 8.

It can be seen from Figure 8 that the MSE of the proposed algorithm is significantly lower than that of other comparison algorithms, especially better than that of the linear detection algorithm of reference [11]. Based on the linear detection algorithm, the neural network is used to compensate for the lack of channel estimation, which is closer to the real channel distribution characteristics. Reference [16] incorporated parallel iteration on the basis of linear detection, and MSE of detection result is reduced, but its data learning ability is somewhat weaker than that of deep learning algorithms. Reference [13] used the iterative precoding algorithm to achieve MIMO signal detection, and its detection accuracy is high. When SNR is 8 dB, its MSE is lower than 0.4. However, the influence of parameters in the deep learning algorithm and the interference of iteration errors are not fully considered, so the detection effect of the proposed algorithm is better. The proposed algorithm uses designed IMPD detector for MIMO signal detection and increases the correction factor and parameter training to reduce detection error. When SNR is 10 dB, its MSE is lower than 0.1, which can meet the requirements of actual environment.

## 5. Conclusion

Massive MIMO technology has become one of key technologies of 5G communication systems due to its high spectrum utilization and link reliability. However, as the number of antennas in the massive MIMO system increases, signal detection will face the challenge of high computational complexity. To this end, this paper proposes a 5G massive MIMO signal detection algorithm based on deep learning. Besides, the sMPD algorithm is used to optimize the network parameters of DNN, and the MIMO system model based on neural network is constructed. The trained DNN detector learns to process the transmission signal to achieve accurate decoding and detection of 5G massive MIMO signal. Experimental results based on TensorFlow deep learning framework show that

1. The DNN detector designed based on the sMPD algorithm has better detection performance and reduces BER through the iterative optimization of correction factor and network parameters. Moreover, the detection performance advantage is obvious.
2. The proposed algorithm builds the MIMO system with the help of neural network learning advantages and uses batch training and dropout to improve the generalization ability of the model, which can accurately and efficiently realize signal detection. When SNR is 10 dB, its BER and MSE are lower than 0.005 and 0.1, respectively.

Since the algorithm in this paper is proposed under the assumption that the channel environment is in an ideal state, the interference of some objective factors is ignored. Further, in-depth research is needed for more nonideal channel environments and realistic system scenarios. In addition, all the proposed improved algorithms only consider the signal detection problem itself, without considering the communication error rate performance that combines it with channel estimation, channel coding, and other issues.

## Figures and Tables

**Figure 1:** Estimation scenario of large-scale MIMO uplink channel.

**Figure 2:** MIMO system model based on neural network.

**Figure 3:** Flow process of data flow.

**Figure 4:** Structure of IMPD detector.

**Figure 5:** Performance comparison between deep learning and linear detection algorithms.

**Figure 6:** Performance comparison between deep learning and belief propagation decoding algorithms.

**Figure 7:** Detection performance comparison of different algorithms.

**Figure 8:** MSE curves of different algorithms.

**Table 1:** MPD diagram model and DNN structure.

MPD	DNN

Node	Neuron
Send signal **x**	Input data *x*
Receive signal **y**	Output data *y*
The *k*-th iteration	The *k*-th hidden layer
Confidence message	Hidden layer information
Data update rules	Hidden relationship of each layer
Correction factor	Parameter *ϖ*

**Table 2:** Simulation parameters.

Parameter	Value

Pilot sequence length	55
Number of base station antennas *M*	100
Signal-to-noise ratio (dB)	10
Number of users *N*	50

## Data Availability

The data used to support the findings of this study are included within the article.
